# Early Warning and Clinical Epidemiological Characteristics of Lung Injury in the Treatment of Infectious *Staphylococcus aureus* Sepsis by Vancomycin Based on Adaptive Niche Genetic Algorithm and Pulmonary Ultrasound Images

**DOI:** 10.1155/2022/3387212

**Published:** 2022-03-07

**Authors:** Xue Huang, Nan Wang, Ningjie Duanmu, Li Fu

**Affiliations:** Department of Emergency, Kunming Yan'an Hospital, Kunming 650000, Yunnan, China

## Abstract

Adaptive niche genetic algorithm (ANGA) and lung ultrasound were combined, the death warning mathematical model was established for patients with sepsis-lung injury, and the epidemiological characteristics were analyzed to explore the efficacy of Vancomycin in the treatment of sepsis-lung injury. First, 88 sepsis patients with lung injury were selected as the research objects. General clinical data and pulmonary ultrasound results were collected. On this basis, epidemiological analysis was carried out, and the death warning model of patients with sepsis-lung injury was established based on ANGA algorithm. Then, the total cure rate, *Staphylococcus aureus* (SA) clearance rate, methicillin-resistant SA (MRSA) clearance rate, and the incidence of adverse reactions after intravenous infusion of Vancomycin were analyzed. The results showed that the ANGA mathematical model combined with the random forest (RF) classifier proposed had better classification effect and robustness relative to the traditional principal component analysis and NGA. The early warning accuracy of the proposed ANGA + RF mathematical model was higher than 95% in contrast to that of the APACHE-II score and the SOFA score. Compared with patients in the severe group, the MRSA infection rate and the levels of procalcitonin (PCT), C-reactive protein (CRP), and activated partial thromboplastin time (APTT) of SA sepsis-lung injury patients were greatly reduced, while thrombin time (TT) and D-D dimer in the death group were considerably increased (*p* < 0.05), and the PLT level was greatly reduced (*p* < 0.05). In addition, the total cure rate, SA clearance rate, and MRSA clearance rate of Vancomycin-treated SA sepsis-lung injury patients were significantly increased (*p* < 0.05) compared with patients in the conventional treatment control group. However, the probability of adverse reactions was increased notably (*p* < 0.05). ANGA combined with RF classifier can improve the accuracy of death warning in patients with sepsis-lung injury. Vancomycin can effectively eliminate MRSA infection rate in patients with sepsis-lung injury and improve the treatment effect of patients.

## 1. Introduction

Sepsis is the most common disease in Intensive Care Medicine (ICU). Even though clinical anti-infection and other treatment methods have made great achievements, the fatality rate of patients with severe infection is still showing a high trend [1]. Sepsis generally refers to external bacteria that enter the blood system through the body surface or the entrance of infection and then multiply in the body's blood, which spread throughout the body along with the blood circulation and then cause systemic symptoms [2]. When sepsis occurs, the lungs are often the first and most vulnerable organ to attack. Sepsis involves the lungs and is known as sepsis-lung injury, with clinical data showing a mortality rate of 50 to 60 percent. Therefore, in the process of clinical treatment of sepsis, in addition to controlling infection, it is also particularly important to avoid or slow down sepsis-lung injury. SA and MRSA are the most common strains that cause Gram-positive sepsis, and they have a high morbidity and mortality rate [3]. Vancomycin is a highly representative antibacterial drug, which is considered to be the last line of defense against Gram-positive bacterial infections clinically. Vancomycin is used in clinical treatment and has a certain antibacterial effect [4, 5]. However, studies found that long-term use of Vancomycin can cause various adverse reactions in patients and poor clinical effects [6]. In addition, the existing studies on the treatment effect of vancomycin are mostly about the treatment of sepsis alone, and there is almost no study on the treatment of sepsis-lung injury. Therefore, understanding the epidemiological characteristics of patients and analyzing the therapeutic effects of Vancomycin are of great significance for formulating corresponding national health policies and improving the prognosis of patients.

With the rapid progression of information technology and medical technology, the medical field has gradually entered the era of intelligence. Mining valuable information from massive medical data has become a research hotspot in artificial intelligence [7]. Classification is a very important step in the data mining process, which can summarize each sample in the data into a known category. However, there is an increase in the unbalanced data in the medical data, and the unbalanced data will cause the imbalance of the sample category, and then it increases the difficulty of classification [8]. The existing feature selection and classifier construction techniques used for imbalanced data classification and processing have many limitations, and it is difficult to screen and obtain effective feature subsets to construct efficient classifiers [9]. Pulmonary ultrasound has been widely used in the diagnosis of pulmonary diseases and has been included in the routine examination methods in some diseases. It also has a better diagnosis for sepsis-lung injury. Therefore, it is very necessary to add pulmonary ultrasound in the data analysis of sepsis and lung injury. Pulmonary ultrasound is a very important and main data for the current research on data analysis of lung injury in sepsis.

Therefore, in this study, a mathematical model was constructed for feature selection and classification of unbalanced data based on lung ultrasound and ANGA algorithm and applied to the classification and processing of clinical data of patients with sepsis. Subsequently, the clinical epidemiological characteristics of the patients were analyzed, and the clinical effects of Vancomycin in the treatment of patients with SA sepsis were explored. This research aimed to provide a basis for clinical diagnosis and treatment of sepsis and medical research, which was of important theoretical significance and clinical application value.

## 2. Methods

### 2.1. Pulmonary Ultrasound Examination Process

Color ultrasonic instrument was used beside the bed, together with the corresponding linear array probe and ultrasonic probe; according to the patient's specific conditions, lung ultrasound examination was performed. The specific examination process was as follows: the examination range was divided as follows: the half chest was divided into the anterior chest wall, the lateral chest wall, and the posterior chest wall by the axillary front line and the posterior axillary line (PAL), and each chest wall was divided into the upper and lower parts, so that each half chest wall was divided into 6 areas and the whole chest was divided into 12 areas. The highest value of the lung ultrasound scoring standard was used as the record value to record the score of each lung region. The sum of the scores of the 12 regions was the lung ultrasound score value. Each lung ultrasound examination was recorded in the lung ultrasound scoring table, and the lung ultrasound score value was calculated. The pulmonary ultrasound score value was the sum of the 12 chest zoning scores, and the score was between 0 and 36 points. The minimum score of 0 represented the ventilation of normal lung tissue, and the ratio of air to water was not abnormal. The highest score was 36, indicating severe consolidation of lung tissue and white lung.

### 2.2. Establishment of Early Warning Model of Sepsis-Lung Injury Based on ANGA Algorithm

Genetic algorithm (GA) is prone to phenomena such as prematurity in the feature selection of medical data. Niche genetic algorithm (NGA) introduces niche based on GA algorithm, which increases the diversity of population evolution and improves the efficiency of feature search [10]. However, the NGA algorithm needs to select good individuals randomly or select good individuals through a control function. Inappropriate individuals or functions will interfere with NGA algorithm, make lack of diversity, and lead to local convergence problems [11]. Therefore, it is proposed to use ANGA to construct the mathematical model of death warning for patients with sepsis, and the implementation process of the ANGA algorithm is as follows.

#### 2.2.1. Calculation of Fitness

Assuming that the size of the initial population is *M* and 2 × *M* individuals are randomly generated, the fitness function is used to calculate the fitness of an individual, and the reciprocal of the sum of squares of the data error obtained by the classifier is used as the fitness function. Then, the mathematical expression is as follows.

(1) $$\begin{array}{c} f\left(x\right)=\frac{1}{\sum_{i=1}^{n}{\left(t_{p}^{i}-t_{a}^{i}\right)}^{2}}. \end{array}$$

In equation (1), *t*_*p*_^*i*^ is the predicted value, *t*_*a*_^*i*^ is the actual value, and *n* is the number of samples.

#### 2.2.2. Niche Elimination Operation

The niche elimination operations are mainly divided into the following steps: (a) adaptive setting of distance parameters, including calculation of distance between individuals and adaptive survival distance; (b) self-adaptive setting of the number of excellent individuals, and the number of individuals *M*_(*t+*1)_ being calculated; (c) the adaptive setting of the population size, and the optimal initial individual *M*_*t*_ being finally obtained. The specific operation process is shown in Figure 1.

#### 2.2.3. Adaptive Crossover and Mutation

When the probability of crossover and mutation is too low, it will cause the algorithm to fall into a local optimal solution. If the probability is too large, however, it will cause problems such as instability of the algorithm and difficulty in convergence. The calculation equations for the probability of adaptive crossover and mutation are as follows.

(2) $$\begin{array}{c} p_{c}=\left\{\begin{array}{cc} p_{c1}-\frac{p_{c1}-p_{c2}}{f_{\max}-f_{\text{avg}}}\left(f\prime -f_{\text{avg}}\right), & f\prime \geq f_{\text{avg}},\\ p_{c1}, & f\prime <f_{\text{avg}}, \end{array}\right. \end{array}$$

(3) $$\begin{array}{c} p_{m}=\left\{\begin{array}{cc} p_{m1}-\frac{p_{m1}-p_{m2}}{f_{\max}-f_{\text{avg}}}\left(f-f_{\text{avg}}\right), & f\geq f_{\text{avg}},\\ p_{m1}, & f<f_{\text{avg}}. \end{array}\right. \end{array}$$

In equations (2) and (3), *f*_max_ is the maximum fitness of the group, *f*_avg_ is the average fitness of the group, *f′* is the greater fitness among the crossover individuals, *f* is the fitness of the variant individual, *p*_*c*_ is the individual crossover probability, and *p*_*m*_ is the probability of individual variation.

#### 2.2.4. Elimination Operation of Niche

The operation of Step II is performed on the new group obtained in the previous step to obtain the optimal individual.

#### 2.2.5. Convergence Judgment of the Algorithm

When the algorithm does not meet the convergence condition, the group generated in the previous step is regarded as the next-generation group, and go to step III. If the algorithm satisfies the convergence condition, the final selected feature is output.

### 2.3. Data Collection of Patients with Sepsis

A total of 88 patients with sepsis and lung injury admitted to hospital from January 2016 to September 2020 were selected as the research subjects. There were 54 male patients and 34 female patients, with an average age of 55.3 ± 11.3 years. Patients included in the study must meet the diagnostic criteria for sepsis-lung injury, and all patients were included only once. The day when the patient was diagnosed with sepsis-lung injury and included in the study was defined as the first day, and data on the patient's clinical characteristics, basic medical history, etiology, treatment measures, and lung ultrasound were collected. The Acute Physiology and Chronic Health Evaluation II (APACHE II) [12] and Sequential Organ Failure Assessment (SOFA) scoring were performed on the first day of the included study [13]. This study obtained the informed consent of patients and their families, who had signed the informed consent forms in strict accordance with relevant regulations. This study had been approved by the Ethics Committee of hospital.

Sepsis was defined as suspected infection or meeting two or more systemic inflammatory response syndrome (SIRS) indicators at the same time. SIRS diagnostic criteria were as follows: (i) core body temperature >36.0°C or <38.0°C; (ii) heart rate >90 beats/min; (iii) respiration rate >20 beats/min, or carbon dioxide partial pressure <32 mmHg, etc.; (iv) white blood cell count >12.0 × 10^9^/L or <4.0 × 10^9^/L, or immature cells >10%. Sepsis-lung injury refers to lung dysfunction on the basis of sepsis.

### 2.4. Operating Parameters of a Mathematical Model for Early Warning of Sepsis-Lung Injury

According to the results on the 28th day, the patient data were classified into negative (no death at 28 days) and positive (death at 28 days) groups. The initial population size of the model was set to 90, and the value of *N* in the memory pool was 30. According to the number of original features of the sample, the length of the individual's gene encoding was set to 75, and the individual's gene location values were “1” and “0”, respectively. “1” indicated that the feature participated in the construction of the model, and “0” indicated that the feature did not participate in the construction of the model. The maximum evolution algebra was set to 100. When the algorithm reached the set value of the maximum evolution algebra, the operation ended.

### 2.5. Evaluation Parameters of the Mathematical Model for Early Warning of Sepsis-Lung Injury

NGA and ANGA algorithms were used to select the characteristics of patient data. In addition, principal component analysis (PCA) was also introduced for special medical treatment. Furthermore, RF, support vector machine (SVM), BP neural network (BPNN), and nearest neighbor algorithm (KNN) were employed for data classification. The execution times of different algorithms were 100 times, and the performance of the algorithm was evaluated regarding the classification accuracy, the number of features, the area under the ROC curve (AUC), and the robustness of the algorithm.

### 2.6. Vancomycin for Treating SA Infection Sepsis-Lung Injury

The patients with sepsis-lung injury who were diagnosed with SA infection were selected for follow-up research, and the patients were randomly rolled into two groups. Patients in the control group received only conventional treatment, while patients in the observation group were given intravenous drip of 0.5 g Vancomycin. The treatment was performed every 8 hours, and the continuous treatment was 7 days as a course of treatment, with a total of 2 courses of treatment.

### 2.7. Clinical Efficacy Evaluation Index

The clinical cure rate of the patient was calculated after the treatment and after the follow-up. The total cure rate of the patients in microbiology after the follow-up was analyzed. In addition, the clearance rate of SA and MRSA after treatment was counted, so did the adverse reactions of patients during the treatment.

### 2.8. Statistical Analysis

Continuous variables conforming to normal distribution were represented by mean plus or minus standard deviation, and dichotomous variables were represented by frequency (percentage). The experimental data were tested by independent sample *t* test or one-way ANOVA analysis of variance, and the test method was selected according to the actual comparison. The survival probability of patients with different disease levels was estimated and analyzed by Kaplan Meier. All statistical analyses were performed using SPSS 19.0, and *p* < 0.05 was considered statistically significant.

## 3. Results

### 3.1. Display of Pulmonary Ultrasound Data of Typical Cases

The pulmonary ultrasound data of a typical case were shown in Figure 2. (a) 1 ultrasound score of line B, 1 point. (b) 2 B-lines ultrasound score, 2 points; (c) fusion B-line ultrasound score, 1 + 2 + 3/2 = 3 points; (d) the fusion B-line ultrasound score (2 + 4)/(1 + 2 + 3 + 4) = 6 points; (e) white lung ultrasound score, 10 points; (f) the ultrasonographic score of subpleural consolidation, 10 points. In the specific scoring process, the scores of each part are added according to the actual situation of the patients to evaluate the pulmonary lesions of the patients.

### 3.2. Test Results of the Mathematical Model for Early Warning of Sepsis-Lung Injury

#### 3.2.1. Comparison of Classification Performance of Mathematical Models

The difference between the classification accuracy of different feature selection mathematical models was compared under different classifiers, and the results were shown in Figure 3. Before feature selection (Origin), the average classification accuracy of RF, SVM, BPNN, and KNN classifiers was all the lowest. The classification accuracy after feature selection using different mathematical models was notably improved. The classification accuracy of the PCA and NGA mathematical models under different classifiers was basically similar, while the classification accuracy of the ANGA mathematical model was obviously the highest.

The difference between the classification of AUC averages of different feature selection mathematical models under different classifiers was compared, and the results were shown in Figure 4. After PCA, NGA, and ANGA mathematical models were adopted for feature selection, the classification of AUC averages of the PCA and NGA mathematical models was basically similar, while the average AUC of the ANGA mathematical model was obviously the highest.

The difference between the number of feature subsets selected by different mathematical models was compared in Figure 5. The decibels of PCA, NGA, and ANGA models had 20 ± 1, 23 ± 2, and 7 ± 1 feature subsets under RF classifier, respectively. The decibels of PCA, NGA, and ANGA models under SVM classifier had 25 ± 2, 20 ± 0.5, and 15 ± 1.2 feature subsets, respectively. The decibels of PCA, NGA, and ANGA models had 17 ± 2, 22 ± 0.5, and 14 ± 1.5 feature subsets under BPNN classifier, respectively. PCA, NGA, and ANGA models had 22 ± 3, 18 ± 2.2, and 11 ± 1.4 feature subsets under KNN classifier, respectively.

#### 3.2.2. Comparison of the Robustness of Mathematical Models

The differences among the GA, NGA, and ANGA mathematical models converging to obtain the global optimal solution under different iteration times were compared, and the results were shown in Figure 6. GA algorithm was iterated to 4 times, NGA algorithm was iterated to 7 times, and ANGA algorithm was iterated to 10 times to converge to obtain the global optimal solution. Obviously, ANGA algorithm had the best global optimal solution ability in contrast to GA and NGA algorithms.

The differences of the convergence speeds of different mathematical models were analyzed in Figure 7. The GA algorithm converged in the 57th generation, the NGA algorithm converged in the 45th generation, and the ANGA algorithm converged with the 21st generation. ANGA algorithm had a faster convergence speed versus that of GA and NGA algorithms.

### 3.3. Data Distribution of Epidemiological Characteristics of Patients with Sepsis-Lung Injury

Clinical treatment data of patients with sepsis-lung injury were collected, and the characteristic data was normalized. The characteristic data were classified according to positive and negative, and the distribution of characteristic values of different data was compared and analyzed. The changes between different clinical data of patients were analyzed first, and the results were shown in Figure 8. The changes in the characteristic distribution of age, creatinine, urea nitrogen, platelets, mean arterial pressure, and respiratory frequency of positive and negative patients were not very obvious. With the increase of the age of patients with sepsis-lung injury, the APACHE-II score and SOFA score of patients showed a gradual increase trend, and the mortality rate of patients also gradually increased. In addition, about 15% of the negative patients were found to be infected with Gram-positive bacteria, and about 30% of the patients were infected with Gram-negative bacteria. Moreover, about 12% of the positive patients were infected with Gram-positive bacteria, and about 36% of patients were infected with Gram-negative bacteria. However, it was difficult to diagnose the patient's condition using a single clinical data.

### 3.4. Early Warning Results of Sepsis-Lung Injury

APACHE-II score is the most commonly used clinical ICU scoring system, and SOFA score can describe the characteristics of organ dysfunction and failure. The APACHE-II score, SOFA score, and the performance difference of the ANGA mathematical model combined with the RF classifier proposed for patient prognosis prediction were compared, and the results were shown in Figure 9. The accuracy and AUC value of the proposed ANGA + RF algorithm for predicting patient prognosis were dramatically superior to APACHE-II score and SOFA score.

### 3.5. Treatment Effect of Patients with SA Sepsis-Lung Injury

According to the results of pathogenic bacteria culture in clinical patients, the clinical data of 107 patients with SA sepsis-lung injury were extracted for analysis, and the epidemiological differences between the survival group and the death group were compared in Table 1. Compared with the survival group, the MRSA infection rate and the levels of procalcitonin (PCT), C-reactive protein (CRP), activated partial thromboplastin time (APTT), thrombin time (TT), and D-D dimer in the death group were remarkably increased (*p* < 0.05), while the PLT level was greatly reduced (*p* < 0.05). There was no considerable difference between the two groups of patients in gender, age, basic medical history, and nosocomial infection rate (*p* > 0.05).

The surviving patients were randomly divided into a control group (*n* = 39) and an observation group (*n* = 44) and were given conventional treatment and Vancomycin treatment, respectively. The difference between the two groups of patients was compared in terms of the treatment effect, and the results were shown in Table 2. The total cure rate, SA clearance rate, and MRSA clearance rate of the observation group increased greatly in contrast to control group (*p* < 0.05). Moreover, the incidence of adverse reactions in the observation group was also remarkably increased (*p* < 0.05).

## 4. Discussion

Severe infection is a common problem that affects the life safety of patients clinically, and the incidence of severe infection is showing an increasing trend year by year. However, the current diagnostic criteria for severe infections are not consistent in the world [14]. With the clinical use of antibacterial drugs, human body has gradually developed resistance to antibacterial drugs, which has led to an increasing trend in hospital and community infection rates year by year. SA and *Staphylococcus epidermidis*-based Gram-positive bacterial infections are the most common [15, 16].

The mining of valuable information in clinical medical data is of great significance for improving treatment measures and improving the treatment effect of patients. Faced with unbalanced data, it is necessary to perform feature selection first and then use the classifier to perform feature classification processing [17]. GA is currently the most common feature selection algorithm, but the population change in the evolution process is relatively single. The algorithm is prone to premature and slow convergence, and it is difficult to obtain the global optimal feature combination [18, 19]. In addition, pulmonary ultrasound plays an important role in the diagnosis of pulmonary diseases, and it also has a good diagnostic effect for sepsis-lung injury. Therefore, this research is based on NGA algorithm and lung ultrasound, and ANGA was proposed, which combined different classifiers to classify the data of sepsis-lung injury patients. The results showed that the accuracy of the proposed ANGA algorithm for data classification was significantly improved compared to the prefeature selection, the PCA algorithm, and the NGA algorithm. Robustness is also one of the important indicators of the evaluation algorithm. Therefore, the convergence of different mathematical models was compared, and the results showed that the convergence performance of the ANGA algorithm was better than that of GA and NGA algorithms.

In the clinical diagnosis and treatment of sepsis-lung injury, age, creatinine, urea nitrogen, platelets, mean arterial pressure, and respiratory rate are the most commonly used characteristic data [20]. Among them, creatinine is used to indicate changes in the patient's renal function, and its decrease is one of the manifestations of exacerbation of sepsis-lung injury [21]. In addition, decreased platelet levels and decreased urea nitrogen levels are all signs of exacerbation of sepsis-lung injury [22]. In this work, the differences in the characteristic distribution of the above-mentioned indicators were compared between the sepsis-lung injury patients and the surviving patients. It was found that the difference in the characteristic distribution of the above-mentioned indicators between the two groups of patients was not obvious. In addition, as the age of patients with sepsis-lung injury increased, the fatality rate, APACHE-II score, and SOFA score all showed a gradually increasing trend [23]. The above results showed that the use of a single characteristic index for early warning of the prognosis of patients with sepsis-lung injury was not excellent. Subsequently, the effects of APACHE-II score, SOFA score, and ANGA mathematical model in predicting patient death were compared. The results showed that the classification accuracy of APACHE-II score and SOFA score was only about 60%, while the classification accuracy of the ANGA mathematical model was as high as 90%.

To further evaluate the clinical efficacy of Vancomycin in patients with SA sepsis and lung injury, supplementary measures were selected to evaluate the difference in peripheral blood coagulation between surviving and dead patients. SA is the first pathogen causing sepsis-lung injury, which accounts for about 15% of all pathogens [24]. Studies confirmed that the mortality rate of patients with SA sepsis-lung injury can reach about 40% clinically [25]. MRSA is more likely to appear in migration in contrast to methicillin-sensitive bacteria, and MRSA is an independent risk factor for death from SA bloodstream infection [3]. The results showed that there were significant differences in PLT, APTT, TT, and D-D dimer between the SA sepsis-lung injury survival group and the death group. PLT reflects the patient's exogenous coagulation ability, while APTT and TT reflect the patient's endogenous coagulation ability. D-D dimer is a degradation product of cross-linked fibrin, which reflects the hypercoagulable state in the body [26–28]. It was found that the PLT level of patients with SA sepsis-lung injury in the death group was reduced, and APTT, TT, and D-D dimer were obviously increased, indicating that the decrease of patient's blood coagulation ability developed the disease. Moreover, the total cure rate, SA clearance rate, and MRSA clearance rate of Vancomycin treatment of surviving SA sepsis-lung injury patients were remarkably improved, but the probability of adverse reactions in patients was greatly increased.

## 5. Conclusion

Lung ultrasound and ANGA algorithm were combined, a warning mathematical model was established for patients with sepsis-lung injury, and its early warning effect was compared with other characteristic indicators. Then, the clinical efficacy of Vancomycin in the treatment of SA sepsis-lung injury was analyzed. The accuracy of the early warning mathematical model based on ANGA and pulmonary ultrasound for patient classification was significantly better than other indicators. Vancomycin to treat patients with SA sepsis-lung injury can improve the clinical treatment effect of patients, but it was easy to increase the adverse reaction rate. However, only the clinical efficacy of Vancomycin in the treatment of SA sepsis-lung injury was analyzed in this work. In recent years, many studies found that linezolid had excellent effects in the treatment of such diseases. Therefore, it is necessary to further find effective drugs for the treatment of SA sepsis-lung injury in the follow-up. To sum up, this study provides a reference for improving the clinical treatment effect of SA sepsis-lung injury.

## Figures and Tables

**Figure 1:** Niche elimination operation process. *Note*. *M* is the number of groups. *x*_*i*_ and *x*_*j*_ are two individuals in the current population. *t* represents algebra. SD is the degree of individual similarity. SD(*x*_*i*_, *x*_*j*_)=∑_*k*=1_^*a*^num(*x*_*ik*_==*x*_*jk*_)/*a*, where *a* is the number of individuals. MSD is the average similarity between the target individual and other individuals. MSD=∑_*j*=*j*+1_^*M*^SD(*x*_*i*_, *x*_*j*_)/*a* · (*M* − 1). *M*_(*t*)_ is the population size of the *t* generation.

**Figure 2:** Display of pulmonary ultrasound data of typical cases.

**Figure 3:** Comparison of classification accuracy of different mathematical models.

**Figure 4:** Comparison of mean AUC of different mathematical models.

**Figure 5:** Comparison of the number of feature subsets selected by different mathematical models.

**Figure 6:** Comparison of convergence of different mathematical models.

**Figure 7:** Comparison of the average evolutionary algebra of convergence of different mathematical models.

**Figure 8:** Distribution of characteristic data of patients with sepsis-lung injury.

**Figure 9:** Comparison of prediction performance of different methods.

**Table 1:** Basic information of patients with SA sepsis-lung injury.

Item	Survival group (*n* = 83)	Death group (*n* = 24)	Statistics	*p*
Male (*n*/%)	44/53.0	13/54.2	1.339	0.286
Age (years old)	35.5 ± 5.7	36.1 ± 4.9	1.297	0.263
Basic medical history (*n*/%)	18/15.7	6/25.0	1.263	0.255
Nosocomial infection rate (*n*/%)	18/15.7	6/25.0	1.263	0.255
MRSA (*n*/%)	18/15.7	19/79.2	38.991	0.000
PCT (*μ*g/L)	3.7 ± 1.3	13.1 ± 5.2	5.778	0.000
CRP (mg/L)	37.6 ± 10.6	88.3 ± 11.9	5.989	0.000
PLT (×10^9^/L)	131.5 ± 26.7	49.8 ± 13.3	6.728	0.000
PDW (fL)	12.5 ± 5.6	14.7 ± 2.8	4.391	0.000
APTT (s)	32.5 ± 6.7	46.2 ± 7.0	6.262	0.000
TT (s)	15.2 ± 3.1	18.9 ± 6.3	5.784	0.000
D-D dimer (mg/L)	2.6 ± 1.7	10.6 ± 5.9	6.397	0.000

**Table 2:** Evaluation of treatment effect of patients.

Item	Control group (*n* = 39)	Observation group (*n* = 44)	Statistics	*p*
Total cure rate (*n*/%)	10/25.6	32/72.7	5.559	0.000
SA clearance rate (*n*/%)	3/7.7	40/90.9	6.687	0.000
MRSA clearance rate (*n*/%)	3/7.7	38/86.4	6.739	0.000
Adverse reaction rate (*n*/%)	2/5.1	13/29.5	5.893	0.000

## Data Availability

The data used to support the findings of this study are available from the corresponding author upon request.
